# Determination of critical epitope of PcMab-47 against human podocalyxin

**DOI:** 10.1016/j.bbrep.2018.04.003

**Published:** 2018-04-24

**Authors:** Shunsuke Itai, Shinji Yamada, Mika K. Kaneko, Yukinari Kato

**Affiliations:** a Department of Antibody Drug Development, Tohoku University Graduate School of Medicine, 2-1 Seiryo-machi, Aoba-ku, Sendai, Miyagi 980-8575, Japan; b New Industry Creation Hatchery Center, Tohoku University, 2-1, Seiryo-machi, Aoba-ku, Sendai, Miyagi 980-8575, Japan

**Keywords:** mAb, monoclonal antibody, SCC, squamous cell carcinoma, DMEM, Dulbecco's Modified Eagle's Medium, EDTA, ethylenediaminetetraacetic acid, BSA, bovine serum albumin, PBS, phosphate-buffered saline, FBS, fetal bovine serum, DAB, 3,3-diaminobenzidine tetrahydrochloride, Podocalyxin, PODXL, Epitope mapping, Monoclonal antibody, Oral cancer

## Abstract

Podocalyxin (PODXL) is a type I transmembrane protein, which is highly glycosylated. PODXL is expressed in some types of human cancer tissues including oral, breast, and lung cancer tissues and may promote tumor growth, invasion, and metastasis. We previously produced PcMab-47, a novel anti-PODXL monoclonal antibody (mAb) which reacts with endogenous PODXL-expressing cancer cell lines and normal cells independently of glycosylation in Western blot, flow cytometry, and immunohistochemical analysis. In this study, we used enzyme-linked immunosorbent assay (ELISA), flow cytometry, and immunohistochemical analysis to determine the epitope of PcMab-47. The minimum epitope of PcMab-47 was found to be Asp207, His208, Leu209, and Met210. A blocking peptide containing this minimum epitope completely neutralized PcMab-47 reaction against oral cancer cells by flow cytometry and immunohistochemical analysis. These findings could lead to the production of more functional anti-PODXL mAbs, which are advantageous for antitumor activities.

## Highlights

• PODXL is involved in cancer growth, invasion, and metastasis.
• PcMab-47 mAb against PODXL shows high ADCC/CDC and antitumor activities.
• PcMab-47 epitope was determined to be Asp207, His208, Leu209, and Met210.
• A blocking peptide completely neutralized PcMab-47 reaction by FCM and IHC.

## 1 Introduction

Podocalyxin (PODXL) is a type I transmembrane protein, which is highly glycosylated and has a molecular weight of 150,000–200,000 [1], [2], [3], [4], [5]. PODXL expression has been reported in several human cancers, including oral [6], breast [7], and lung cancer [8], [9] and leads to tumor growth, invasion, and metastasis [7], [10]. Several studies have developed anti-PODXL monoclonal antibodies (mAbs) [11], [12].

We previously produced a novel anti-PODXL mAb, PcMab-47 (IgG_1_, kappa) [13]. PcMab-47 reacts with endogenous PODXL-expressing cancer cell lines and normal cells independently of glycosylation in Western blot, flow cytometry, and immunohistochemical analysis. We engineered PcMab-47 into 47-mG_2a_, a mouse IgG_2a_-type mAb, to add antibody-dependent cellular cytotoxicity (ADCC). We further developed 47-mG_2a_-f, a core fucose-deficient type of 47-mG_2a_, to augment its ADCC. Immunohistochemical analysis of oral cancer tissues using PcMab-47 and 47-mG_2a_ revealed that the latter stained oral squamous cell carcinoma (OSCC) cells in a cytoplasmic pattern at a much lower concentration than the former. *In vitro* analysis showed that 47-mG_2a_-f exhibited a much stronger ADCC than 47-mG_2a_ against OSCC cells. *In vivo* analysis revealed that 47-mG_2a_-f, but not 47-mG_2a_, exerted an antitumor activity in SAS and HSC-2 xenograft models at a dose of 100 μg/mouse/week administered three times. Although 47-mG_2a_ and 47-mG_2a_-f exerted antitumor activities in HSC-2 xenograft models at a dose of 500 μg/mouse/week administered twice, 47-mG_2a_-f showed a higher antitumor activity than 47-mG_2a_. These results suggested that a core fucose-deficient anti-PODXL mAb could be useful for antibody-based therapy against PODXL-expressing OSCCs. Although engineered mAbs of PcMab-47 show high antitumor activities against cancer cells, the critical epitope of PcMab-47 remains to be identified.

In this study, we clarified the binding epitope of PcMab-47 using enzyme-linked immunosorbent assay (ELISA), flow cytometry, and immunohistochemistry.

## 2 Materials and methods

### 2.1 Cell lines

CHO-K1 was obtained from the American Type Culture Collection (ATCC, Manassas, VA). SAS (oral squamous carcinoma cell line from tongue) was obtained from the Japanese Collection of Research Bioresources Cell Bank (Osaka, Japan). CHO-K1 cells were transfected with PA-tagged PODXL deletion mutant plasmids using Lipofectamine LTX (Thermo Fisher Scientific Inc., Waltham, MA). PODXL deletion mutants were cultured in an RPMI 1640 medium (Nacalai Tesque, Inc., Kyoto, Japan), and SAS was cultured in Dulbecco's Modified Eagle's Medium (DMEM; Nacalai Tesque, Inc.), supplemented with 10% heat-inactivated fetal bovine serum (Thermo Fisher Scientific Inc.), 100 units/ml penicillin, 100 μg/ml streptomycin, and 25 μg/ml amphotericin B (Nacalai Tesque, Inc.), and incubated at 37 °C in a humidified atmosphere of 5% CO_2_ and 95% air.

### 2.2 Plasmid preparation

The cDNA encoding the full-length open reading frame (ORF) of PODXL was obtained by PCR using cDNA derived from the LN229 cell line (ATCC) as a template. Appropriate oligonucleotides were used as primers to make each deletion mutants. PCR products were subcloned into pCAG vector (FUJIFILM Wako Pure Chemical Industries Ltd., Osaka, Japan) with signal sequence and PA tag using the In-Fusion PCR Cloning kit (Takara Bio, Inc., Shiga, Japan). All amino acid number were consistent with the NCBI Reference Sequence, NP_005388.2.

### 2.3 Enzyme-linked immunosorbent assay (ELISA)

Synthesized PODXL peptides (PEPScreen; Sigma-Aldrich Corp., St. Louis, MO) were immobilized on Nunc Maxisorp 96-well immunoplates (Thermo Fisher Scientific Inc.) at 1 μg/ml for 30 min. After blocking with SuperBlock T20 (PBS) Blocking Buffer (Thermo Fisher Scientific Inc.), the plates were incubated with purified PcMab-47 (1 μg/ml), followed by a 1:2000 dilution of peroxidase-conjugated anti-mouse IgG (Agilent Technologies Inc., Santa Clara, CA). The enzymatic reaction was conducted using 1-Step Ultra TMB-ELISA (Thermo Fisher Scientific Inc.). Optical density was measured at 655 nm using an iMark microplate reader (Bio-Rad Laboratories, Inc., Berkeley, CA). These reactions were performed at 37 °C with a total sample volume of 50–100 μl.

### 2.4 Flow cytometry

Cells were harvested after brief exposure to 0.25% trypsin/1 mM ethylenediaminetetraacetic acid (EDTA; Nacalai Tesque, Inc.). After washing with 0.1% bovine serum albumin in PBS, the cells were treated with PcMab-47 (1 μg/ml) or PcMab-47 (1 μg/ml) plus peptides (1 μg/ml) for 30 min at 4 °C, followed by treatment with Alexa Fluor 488-conjugated anti-mouse IgG (1:1000; Cell Signaling Technology, Inc., Danvers, MA). Fluorescence data were acquired using the Cell Analyzer SA3800 (Sony Corp., Tokyo, Japan).

### 2.5 Immunohistochemical analyses

Histological sections of 4-μm thickness were directly autoclaved in citrate buffer (pH 6.0; Nichirei Biosciences, Inc., Tokyo, Japan) for 20 min. Sections were then incubated with PcMab-47 (5 μg/ml) or PcMab-47 (5 μg/ml) plus peptides (5 μg/ml) for 1 h at room temperature, treated using an Envision+ kit (Agilent Technologies Inc.) for 30 min. Color was developed using 3,3-diaminobenzidine tetrahydrochloride (DAB; Agilent Technologies Inc.) for 2 min, and counterstained with hematoxylin (FUJIFILM Wako Pure Chemical Industries Ltd.).

## 3 Results and discussion

We previously developed PcMab-47, a novel anti-PODXL mAb which exhibits a high specificity and sensitivity against human PODXL. PcMab-47 was shown to be useful for immunohistochemical analyses using paraffin-embedded tissues [13], [14]. Furthermore, engineered mAbs of PcMab-47 exerted high antitumor activities against cancer cells in mouse xenograft models. Therefore, the determination of the binding epitope of PcMab-47 is critical to further develop a molecular targeting therapy against PODXL.

In this study, eight deletion mutants of PODXL were constructed (Fig. 1A). Stable transfections of PODXL-mutant clones were established on CHO-K1 cells, including dN25 (corresponding to 25–526 amino acids [aa]), dN80 (corresponding to 80–526 aa), dN100 (corresponding to 100–526 aa), dN140 (corresponding to 140–526 aa), dN180 (corresponding to 180–526 aa), dN200 (corresponding to 200–526 aa), dN220 (corresponding to 220–526 aa), and dN300 (corresponding to 300–526 aa). All deletion mutants of PODXL contained an N-terminal PA tag and were analyzed using flow cytometry for the epitope mapping of PcMab-47. NZ-1 (anti-PA tag mAb) detected all deletion mutants of PODXL, including dN25, dN80, dN100, dN140, dN180, dN200, dN220, and dN300 (Fig. 1A, upper panel). In contrast, PcMab-47 did not react with dN220 and dN300 (Fig. 1A, lower panel). These results indicate that the N-terminus of PcMab-47 epitope exists between the 200th and 219th aa. These results are summarized in Fig. 1B.

**Fig. 1:** (A) Flow cytometry using deletion mutants of PODXL. PcMab-47 and anti-PA tag (NZ-1) were treated with deletion mutants of PODXL cells for 30 min at 4 °C, followed by the addition of secondary antibodies. Gray peak, negative control; blue peak, anti-PA tag; red peak, PcMab-47. (B) Schematic illustration of the PcMab-47-epitope.

We next synthesized a series of PODXL peptides such as 180–199 aa, 190–209 aa, 200–219 aa, 210–229 aa, 220–239 aa, and 230–249 aa (Table 1, Fig. 1B). PcMab-47 reacted only with 200–219 aa peptides in ELISA. We synthesized a series of point mutations of PODXL peptides of 200–219 aa (Table 1). PcMab-47 reacted with T200A, P201A, T202A, S203A, S204A, G205A, H206A, K211A, S213A, S214A, S215A, S216A, S217A, T218A, and V219A. PcMab-47 weakly reacted with I212A and did not react with D207A, H208A, L209A, or M210A, indicating that PODXL peptides from the 207th to the 210th aa (_207-_DHLM_−210_ sequence) constitute the critical minimum epitope of PcMab-47.

**Table 1:** Determination of PcMab-47 Epitope by ELISA.

*Peptide*	*Sequence*	*PcMab-47*
180–199	TPHPTSPLSPRQPTSTHPVA	−
190–209	RQPTSTHPVATPTSSGHDHL	−
200–219	TPTSSGHDHLMKISSSSSTV	＋＋＋
210–229	MKISSSSSTVAIPGYTFTSP	−
220–239	AIPGYTFTSPGMTTTLPSSV	−
230–249	GMTTTLPSSVISQRTQQTSS	−
T200A	APTSSGHDHLMKISSSSSTV	＋＋
P201A	TATSSGHDHLMKISSSSSTV	＋＋
T202A	TPASSGHDHLMKISSSSSTV	＋＋
S203A	TPTASGHDHLMKISSSSSTV	＋＋
S204A	TPTSAGHDHLMKISSSSSTV	＋＋
G205A	TPTSSAHDHLMKISSSSSTV	＋＋
H206A	TPTSSGADHLMKISSSSSTV	＋＋＋
D207A	TPTSSGHAHLMKISSSSSTV	−
H208A	TPTSSGHDALMKISSSSSTV	−
L209A	TPTSSGHDHAMKISSSSSTV	−
M210A	TPTSSGHDHLAKISSSSSTV	−
K211A	TPTSSGHDHLMAISSSSSTV	＋＋＋
I212A	TPTSSGHDHLMKASSSSSTV	＋
S213A	TPTSSGHDHLMKIASSSSTV	＋＋
S214A	TPTSSGHDHLMKISASSSTV	＋＋＋
S215A	TPTSSGHDHLMKISSASSTV	＋＋＋
S216A	TPTSSGHDHLMKISSSASTV	＋＋
S217A	TPTSSGHDHLMKISSSSATV	＋＋
T218A	TPTSSGHDHLMKISSSSSAV	＋＋＋
V219A	TPTSSGHDHLMKISSSSSTA	＋＋＋

＋＋＋, OD655 ≧ 0.7; ＋＋, 0.4 ≦ OD655＜0.7; ＋, 0.1 ≦ OD655＜0.4; -, OD655＜0.1.

We further performed a blocking assay using flow cytometry. PcMab-47 reacted with the SAS cell line (Fig. 2). This reaction was completely neutralized by the wild-type peptide (_200-_TPTSSGHDHLMKISSSSSTV_-219_), H206A, and K211A. In contrast, D207A, H208A, L209A, and M210A did not block the reaction of PcMab-47 with SAS, confirming that the (_207-_DHLM_-210_) sequence is a critical epitope of PcMab-47.

**Fig. 2:** (A) Flow cytometry using SAS cells. PcMab-47 (1 μg/ml) and PcMab-47 (1 μg/ml) + wild-type peptide (_200-_TPTSSGHDHLMKISSSSSTV_-219_; 1 μg/ml) were treated with SAS cells for 30 min at 4 °C, followed by the addition of secondary antibodies. Gray peak, negative control; red peak, PcMab-47. (B) Flow cytometry using SAS cells. PcMab-47 (1 μg/ml) + each peptide (1 μg/ml) was treated with SAS cells for 30 min at 4 °C, followed by the addition of secondary antibodies. Gray peak, negative control; red peak, PcMab-47 + each peptide.

Finally, we performed a blocking assay using immunohistochemistry. PcMab-47 reacted with oral cancer tissues (Fig. 3A) and the reaction was completely neutralized by the wild-type peptide (_200-_TPTSSGHDHLMKISSSSSTV_-219_) and H206A. D207A did not block the reaction of PcMab-47, and this confirmed the results of the flow cytometric blocking assays.

**Fig. 3:** (A) Immunohistochemistry using oral cancers. Oral cancer tissues were autoclaved in a citrate buffer for 20 min. Sections were then incubated with PcMab-47 (5 μg/ml), PcMab-47 (5 μg/ml), + wild-type peptide (WT, _200-_TPTSSGHDHLMKISSSSSTV_-219_; 5 μg/ml), PcMab-47 (5 μg/ml) + H206A (5 μg/ml), or PcMab-47 (5 μg/ml), + D207A (5 μg/ml) and treated using an Envision + kit. Color development was performed using 3,3-diaminobenzidine tetrahydrochloride. Sections were then counterstained with hematoxylin. The scale bar represents 100 µm. (B) Schematic illustration of PODXL and the PcMab-47-epitope. The critical epitope of PcMab-47 is _207-_DHLM_-210_. SS, signal peptide; TM, transmembrane; IC, intracellular region.

Taken together, our results indicate that the critical epitope of PcMab-47 is Asp207, His208, Leu209, and Met210. Our findings could lead to the production of more functional anti-PODXL mAbs, which would be advantageous for antitumor effects against PODXL-expressing cancers.
